# Observation on the Effect of Rehabilitative Physical Training on Sports Injuries under Ultrasound Image Examination

This article has been retracted.

**DOI:** 10.1155/2022/9998265

**Published:** 2022-06-29

**Authors:** Lanfeng Wang, Haoyu Wang

**Affiliations:** Gdansk University of Physical Education and Sport, Gdansk, Poland

## Abstract

In order to observe the effect of rehabilitative physical training on sports injuries under ultrasound examination, this study firstly carried out experiments, induction and analysis of ultrasound examination, and evaluation-related content, especially the diagnosis of ultrasound examination in muscle and tendon injuries caused by various reasons. And the clinical application of treatment (clinical research) is reviewed, in order to provide reference data for clinical stage summary. Then, by determining the fasciculation and location of the tendon rupture injury by ultrasound, the clinic can decide whether or not to proceed with surgery. Small Achilles tendon tears only require conservative treatment to avoid the development of complete Achilles tendon rupture. Finally, 26 patients and 10 healthy adults were examined by ultrasonography, and each subject was segmented to examine 11 muscles, including the tongue muscle. The bilateral trapezius, bilateral biceps brachii, bilateral abductor pollicis brevis, bilateral quadriceps femoris, and bilateral tibialis anterior muscles were evaluated by ultrasound and statistical methods. The experimental results show that if the fasciculation of the Achilles tendon injury does not reach more than 3/11, it indicates that no surgical treatment is required; for those with a complete tear of the Achilles tendon, the distance between the broken ends should be further measured in the toe flexion state to evaluate whether surgical treatment is required. It effectively solves the problem of visual diagnosis of sports injuries.

## 1. Introduction

Common clinical imaging diagnostic techniques mainly include X-ray, computed tomography (CT), magnetic resonance imaging (MRI), and ultrasound [1]. In the diagnosis of soft tissue lesions such as muscles and tendons, X-ray examination is difficult to clearly display soft tissue lesions, and the detection sensitivity of early lesions is poor; so, it is not applicable for the diagnosis of such diseases (Figure 1). X-ray examination is more suitable for the detection of abnormal structural changes in bones and joints. CT and MRI have clear advantages in diagnosing the anatomical details of musculoskeletal system, muscles, tendons, and other soft tissue lesions; however, its clinical application is limited by the purchase of equipment in medical institutions, whether the operating physicians have professional skills and experience, etc., there are strict requirements for the indication population. Ultrasonography is widely used in clinical practice because of its advantages of noninvasiveness, simple operation, and quick results. Existing studies have shown that ultrasonography can detect skeletal, muscular system muscles, tendons, joints and superficial soft tissue injuries, and even deep muscle lesions. Ultrasonography can dynamically observe the movement of muscles and tendons in real time [2]. However, both CT and MRI cannot perform real-time dynamic examination, which is the main deficiency in their clinical diagnostic applications.

Computed tomography (CT), magnetic resonance imaging (MRI), and ultrasound can be used to diagnose and treat musculoskeletal disorders, both positive and negative. Compared to CT and MRI, ultrasound is easier for patients to receive and can be transmitted in a hospital for the first time. This is a normal observation. In recent years, new ultrasound technology has increased the benefits of conventional ultrasound treatment and compensated for the inadequacy of imaging, especially in diagnostic and diagnostic procedures: treatment of musculoskeletal disorders. To this end, the author discusses the use of ultrasound in the diagnosis and treatment of bone and bone marrow to provide a summary of medical data [3].

## 2. Literature Review

In my country's competitive sports, “physical rehabilitation training” was formally proposed by Dr. Deshmukh et al., and it belongs to a relatively new discipline, but it does not deny that there is no relevant training in our country before [4]. Bertollo and others believe that in foreign countries, the application of rehabilitation physical training to physical training is relatively tight, the training is more refined, the training institutions are more commercial, there are sports rehabilitators, sports protectionists, and physical trainers in terms of personnel distribution, and these three professional talents play a very important role in the medical treatment and physical training of athletes [5]. Gr Bovi et al. believe that a new definition has been added on the basis of the definition of the concept of physical rehabilitation, which is roughly classified as adding attribution: a highly targeted functional training; adding functional value: enabling athletes who are injured or in poor competitive condition to reduce the risk of injury and improve their competitive status; add specificity: combined with special training, it is beneficial to improve the physical function and physical quality of athletes and help athletes prevent sports injuries; and add key differences: in physical rehabilitation training, rehabilitation is the core, and training is the soul [6]. Kudo-Saito and others believe that individualization and differentiated treatment should be emphasized, the impact of injuries on athletes' physical functions should be understood from training, and training plans should be adjusted in time according to athletes' feedback. Among them, Kudo-Saito et al. believe that rehabilitation physical training belongs to a new comprehensive discipline [7]; Choi et al. believe that it is a training method and belongs to functional training; Liu Dongsen believes that it is a physical training program. The ultimate goal of rehabilitative physical training for athletes is not only to restore basic functions but also to improve physical function and sports performance and return to training ground and competition field. For the stage of acute injury of athletes and local inflammation after surgery, medical rehabilitation must be the main focus, and the rest of the body should be rehabilitative physical training by means of balance training [8]. Haller et al. found that there are various classifications of rehabilitation, classifying rehabilitation from the perspective of physiology, and there are sports system rehabilitation, nervous system rehabilitation, cardiopulmonary function rehabilitation, urinary system function rehabilitation, circulatory function rehabilitation, respiratory system function rehabilitation, digestive system function rehabilitation, reproductive system function rehabilitation, and endocrine system function rehabilitation [9]. Xun et al. found that, according to the stage of sports injury recovery, it can be divided into the following: it includes 4 stages: acute stage of injury, medical rehabilitation period, rehabilitation fitness period, and physical training period. It can be divided into upper extremity, lower extremity, and core area according to the part of injury recovery, which is further divided into muscle injury, ligament injury, fascia injury, muscle key sheath, and joint capsule injury. According to the specific purpose of rehabilitation, it can be divided into functional rehabilitation type, disease prevention type, functional rehabilitation type, core strengthening type, nerve rehabilitation type, muscle group rehabilitation type, balance and joint rehabilitation type, and stretching rehabilitation type of physical training [10]. Guo et al. found that physical fitness is divided into broad and narrow concepts, and generalized physical fitness refers to the physical ability elements stored by the human body in order to adapt to the needs of exercise, which is the performance of the basic ability of human activities. The narrow concept is the synthesis of the special strength system and related qualities that athletes need to complete high-level competition [11]. Traylor et al. divided the concept of physical fitness into physiological aspects and psychological aspects, physiological aspects represent sports performance and adaptability, and mental abilities represent the second manifestation of volitional qualities. Traylor et al. more comprehensively summarized the influence of nature and nurture, the elements of physical fitness, and the core quality in the elements [12].

The author takes the content system of rehabilitative physical training as the research object, from the theoretical basis of rehabilitative physical training, to the concept and principle of the programmatic construction of the content system, and the programmatic construction of the content system of rehabilitative physical training, etc.; to sort out the article, the program is used to construct the system, and the program of the rehabilitation physical training content is reflected through case presentation.

## 3. Research Methods

### 3.1. Ultrasound Examination and Evaluation

#### 3.1.1. Ultrasound Inspection Equipment

The authors used the Mindray M7 Ultrasonic System with 11 MHz linear high-frequency probe, and in all tests, all settings were stored in the factory preset tissue imaging facility, with a magnification of 50 and one seeks depth and breadth for each. Muscles and self are different [13].

Ultrasound was performed on 26 patients and 10 adults for good health, and each study examined 11 muscles, including the tongue, two-sided trapezius, two-sided biceps, two-sided abductor pollicis brevis, two lateral quadriceps, and both anterior tibial. The specific inspection methods are as follows: (1) medullary segment: check the tongue muscle and bilateral trapezius muscle and check the trapezius muscle from the back at the level of the cervical spinous process and the midclavicular line; (2) cervical segment: check bilateral biceps and bilateral abductor pollicis brevis; and (3) lumbosacral segment: check bilateral quadriceps and bilateral tibialis anterior muscles. All subjects were trained by 1 or 2 muscle ultrasound and the inspection by professionals who are proficient in muscle ultrasound technology, and the examiner knows the clinical findings of each subject but is unaware of the final diagnosis of each patient. The tongue and bilateral trapezius muscles were examined in a sitting position, and other muscles were examined in a supine position [14]. During the examination, the subject's muscles remain completely relaxed. With the exception of the trapezius, the rest of the muscles were imaged laterally at the largest diameter with B-mode.

#### 3.1.2. Counting Method of Ultrasonic Beam Flutter

Referring to the method of Tsuji et al. to detect fasciculation by ultrasound, the probe was hit in the middle of the muscle belly of each muscle and observed for 30 seconds, ultrasound-identified fasciculations are unspontaneous twitching of a small part of the muscle, for 0.2 to 0.5 s, observe at least three fasciculations in the same muscle (three identical or independent fasciculations), and detected by ultrasound, and it is recorded as a fasciculation detected. In order to assess whether ultrasound can correctly identify fasciculations, when examining each muscle group, the probe detection area needs to be changed, in order to rule out the problem that the muscle structure itself and the surrounding tissue cannot be evaluated, the fasciculation detection is affected. Record the number and types of observed muscle fasciculations; according to the distribution of fasciculations, the fasciculations are divided into two types: focal and multifocal, and the number of fasciculations in each muscle is calculated separately. For muscles with continuous multifocal fasciculations that are difficult to count, count as a maximum of 30. Patients with suspected ALS and healthy adult controls were tested in the same way, and the number and distribution of muscle fasciculations were recorded.

#### 3.1.3. Ultrasound Beam Score

To differentiate ALS patients from non-ALS patients, an “Ultrasonic fibrillation score” developed, which was determined by the number of muscles seen by fasciculation in the muscle selection by ultrasound. Use the ROC curve to find the most important and measure the sensitivity and specificity of the number of fascicular muscles in a patient to differentiate ALS in non-ALS patients: diagnosis of ALS [15].

#### 3.1.4. Statistical Methods

All data in this study were analyzed using SPSS statistics 22.0. Age, gender, number of muscle fasciculation, and amount of fasciculation detected were compared by ALS group, non-ALS control group, and health control group, and the measurement data are presented as the normal distribution. The measurement data conforming to normal distribution were expressed in the form of mean standard deviation (SD) and comparison of the two groups were designed using the independent model *t*-test; census data were presented at different frequencies, and differences between two or more digits were determined using the Kruskal-Wallis test or the Man-Whitney *U* test. Pearson's chi-square test was used to calculate muscle differences and differences between groups of ALS and non-ALS. ROC regression was used to verify the accuracy of the diagnosis, mark the ROC curve, calculate the area under the curve (AUC), find the optimal cut-off value, and identify the sensitivity and specificity. Spearman correlation analysis was used to filter the relationships between difference and nondifference. Each key test is a two-way test. *P* < 0.05 was considered significant (Table 1).

### 3.2. Distribution of Fasciculations Detected by Ultrasound in Each Group

The classification of muscle fasciculation in the ALS group, the control group, and the health control group was 2.5, 0.6, and 0.3, respectively. The distribution of fasciculation differs between three groups (*P* < 0.001) values [16]. Compared with the disease control group and the health control group, the distribution of muscle fasciculation in the group of ALS patients is constant, and the anatomical distribution is broad, generally living into 2 or more segments, and in the distal and near end and follows the results of electromyography, which showed the patient symptoms and upper and lower motor brain damage. Most patients in the control group had no more than 1 stage of fasciculation, but our results showed 2 stages of fasciculation per patient, and in healthy individuals, distribution of fasciculation is most often affected and involved in 2 segments (Figure 2).

### 3.3. Comparison of Fasciculation Muscle Number and Fasciculation Detection Rate among Groups

The number of fasciculations diagnosed in each of the 11 subgroups in the ALS group, the control group, and the health control group was 6.44, 1.20, and 0.50, respectively, and the numbers of people are very different. Of the three groups, the number of fascial muscles found in the ALS group was higher than that in the disease group and the health control group (*P* < 0.001), and the difference was significant (see Table 2).

As shown in Tables 2 and 3, the overall detection rate of fibrillation in the ALS group, the non-ALS control group, and the health management group was 58.5%, 10.9%, and 4.5%, respectively, according to the Kruskal-Wallis *U* test. The rate of detection of total muscle fasciculation was significantly different in the three groups (*H* = 24.008, *P* < 0.001), and the detection rate of fasciculation in the ALS group was higher than in the non-ALS group and health management committee. Of the 176 muscles in the ALS group, 103 were diagnosed with fasciculation, with the muscles with the highest scores being the right two-headed (81.3%) and the tongue with the lowest scoring (18.8%) item. The muscle segment we tested, the lumbosacral fasciculation muscle, had the highest detection rate. Fasciculation was found in 12 of the 110 muscles in the non-ALS control group, with the most common in the left biceps (30%) and no fasciculation in the three elongated muscles (0). Of the 110 muscles in the healthy adult group, only 5 had fasciculation, with two left head (10%), two right head (10%), right leg muscle (10%), anterior left tibia (10%), and right tibia anterior muscle (10%) [17].

Table 3 shows that the diagnosis of muscle fasciculation differs from the distribution of muscles in an individual in the ALS group, the disease control group, and the health control group, and the high level of fasciculation detection is usually divided into lower extremities (lumbosacral segment): quadriceps femoris and anterior tibial muscle. With the exception of muscle mass, the detection of fasciculation in each muscle of the ALS group was greater than in the health control group, and the right biceps, the right pollicis brevis, and the fourth were as follows. The lower limbs are important square test*P* < 0.001. The difference is significant. The detection rate of ALS muscle fasciculation is generally higher in the control group, but the detection rate of the following three muscle fasciculations does not differ between the two groups, namely, left biceps and left abductor pollicis brevis [18].

In all groups of ALS patients with upper and lower tubercle onset, the detection rate of fasciculation was 60.84% and 48.49%, *P* = 0.376, and the difference was not significant. According to the diagnostic procedure for Awaji ALS, there should be no significant differences in the diagnosis of muscle fasciculation in patients with ALS confirmed and those with ALS outcome and in the study Mann–Whitney*U*detector*P* = 0.302(*P* > 0.05). He met the medical procedure for Avaji.

Spearman's analysis of the relationship between the speed of diagnosis of fasciitis in the ALS group and two diagnoses of ALS (chronic disease, ALSFRS-R) shows that the value of investigation of muscle fasciculation by muscle ultrasound is associated with acute myocardial infarction (ALSFRS). *R* was negative (*r* = 0.501), the results were significant (*P* < 0.05), and the detection rate of ALS fasciculation was independent of infection ((*r*) = 0.014, *P* = 0.960). The results are shown in Table 4.

### 3.4. Accuracy of “Ultrasonic Beam Fibrillation Score” in the Diagnosis of ALS

To help identify ALS patients in the diagnosis and treatment of non-ALS disease and health control groups, we developed “fasciculation scores,” which are defined as muscles with fasciculation detected by muscle ultrasound: 11 bodies. Quantity was as follows. Compared with the control group (0.85 ± 1.531), this score was higher in the ALS group (6.44 ± 2.56), *P* < 0.001, and the difference was significant. The area below the ROC curve was used to measure the further diagnosis of ultrasonic radiation fibrillation scores. The results showed that the area under ROC curve (AUC) was 0.96, AUC > 0.9, with liver biopsy and accuracy.

### 3.5. High Frequency Ultrasound Examination

Closed muscle and tendon injuries are common in clinical practice. For example, the common clinical injuries of fingers, wrist, Achilles tendon, quadriceps tendon, etc. are mostly closed muscle and tendon injuries. Routine ultrasonography fails to identify closed muscles, edema due to muscle, tendon rupture in tendon injuries, hemorrhage, and lymphocytic inflammatory infiltration, hypoechoic images appear due to degeneration and necrosis of damaged tissue or local hypoechoic (calcium deposition) due to disease progression and old lesions, strip hyperechoic (fibrogranular tissue, nodule), etc. or may overlook the scan of the proximal end of the ruptured tendon, resulting in missed diagnosis [19].

Compared with conventional ultrasonography, high frequency ultrasonography can clearly diagnose and evaluate the structural and morphological changes and echoic changes of muscle and tendon injuries, and it can more accurately locate the relationship between the injury site, extent, and surrounding tissues (with or without adhesion), degree (with or without fracture) and whether there is hematoma formation. High-frequency ultrasonography is more sensitive than conventional ultrasonography to detect hidden muscle and tendon lesions. High-frequency ultrasound is better than MRI in resolving the fine structure of muscle and can provide more detailed diagnostic information for clinical practice. Li Jing's study used high-frequency ultrasound (5-10 Hz) to examine 135 patients with calf tendon and muscle injuries, and the results show that high-frequency ultrasonography can detect muscle contusion, tear and tendon injury, and rupture patients and can accurately assess the course (acute, chronic) and degree of disease (partial/complete rupture) [20]. Simple operation, strong repeatability, and high resolution in the diagnosis of lower extremity muscle and tendon injuries and high-frequency ultrasonography can provide clearer and more accurate ultrasonographic images, which can improve the positive rate of clinical diagnosis of lower extremity muscle and tendon injuries. In conclusion, the application of high-frequency ultrasound has advantages in the diagnosis of superficial organ lesions, muscle, and soft tissue damage [21].

Because ultrasonography cannot clearly display the whole picture of blood vessels and the details of anatomical structure, there are certain limitations in the diagnosis of soft tissue tumors. High-frequency ultrasonography was used for the diagnosis of muscular system lesions with high sensitivity (100%). Muscle injury, tumor and inflammatory lesions, tendon rupture, ligamentous fibroma, etc. can show specific changes on high-frequency ultrasonography [22]. Therefore, the author believes that high-frequency ultrasonography can be used for the diagnosis of muscle, tendon injury, hemangioma, and other space-occupying lesions. Because high-frequency ultrasonography can display lesions from multiple sections and orientations, it can dynamically observe hematoma changes, etc., and it can clearly distinguish cystic and solid lesions; so, high-frequency ultrasonography has expanded the application scope of ultrasonography, making ultrasonography more and more widely used in the diagnosis of muscle system injuries and tumors.

## 4. Result Analysis

This study examined the role of muscle ultrasound in the diagnosis of ALS by studying muscle fasciculation. What we have found is that muscle ultrasound detects more muscle mass in patients with ALS, making it easier to diagnose ALS and more effective in diagnosing it. Muscle ultrasound can provide important information about fasciculation in patients with neurological and musculoskeletal disorders. Our study showed that there was a significant difference between the prevalence of fasciculation detected by ultrasound examination of patients with ALS and those suspected of having ALS in patients with ALS and older healthy people. We also demonstrated that muscle ultrasound has a higher sensitivity for the detection of muscle fasciculations in ALS patients and developed a more concise and convenient ultrasound fasciculation score to assist in the diagnosis of ALS; that is, 3 of 11 muscles in each patient were detected. Fasciculation, that is, ultrasound fasciculation reaching 3/11, can be used as a diagnostic marker in ALS patients [23].

Under the guidance of ultrasound, local lesions can be located, guided puncture and auxiliary diagnosis, and tendon lengthening surgery, fenestration surgery can be performed for patients with tendinopathy, and injection therapy can be performed for muscle tear injuries and tendinopathy and interventional therapy for bone, muscle, tendinopathy, or nerve damage [24]. By determining the fasciculation and location of tendon rupture injuries by ultrasound examination, the clinic can decide whether to take surgical treatment of the patient. Small Achilles tendon tears only need conservative treatment to avoid developing into complete Achilles tendon rupture. If the fasciculation of the Achilles tendon injury is less than 3/11 after ultrasound evaluation and statistical evaluation, no surgical treatment is required. For those with a complete tear of the Achilles tendon, it is necessary to further measure the distance between the broken ends in the toe flexion state, in order to evaluate surgical treatment. Visible, through ultrasonography, the diagnosis of tendon injury can provide positive guidance for clinical determination of treatment plan. For the diagnosis of muscle and tendon injury, X-ray has no diagnostic specificity; CT, MRI, etc. have high diagnostic rates, but their clinical application is limited. Ultrasound examination is noninvasive, simple to operate, reproducible, and can quickly obtain diagnostic results. It plays an important role in the diagnosis of muscle and tendon injuries. In clinical practice, more application of ultrasonic fusion imaging technology, in order to do a good job of differential diagnosis, improves the accuracy of diagnosis [25].

## 5. Conclusion

The author conducts experiments, induction, and analysis of the relevant contents of ultrasound examination and evaluation, and the data confirms that ultrasound examination can meet the needs of sports injury visualization. Due to time constraints, the programmatic content system proposed by the author has not found enough practical cases to prove it. The rationality and rigor of the content system programming still need to be further verified in future practice. In future research, quantitative research needs to be carried out according to specific cases to determine more quantitative indicators, in order to confirm the effect of the program of rehabilitative physical training under ultrasound examination. In short, the programming of the content system of rehabilitation physical training under ultrasound examination needs to be further verified in future research and makes the program arrangement more reasonable and scientific.

## Figures and Tables

**Figure 1:** Ultrasonic examination.

**Figure 2:** Anatomical distribution of three groups of muscle fasciculations.

**Table 1:** Demographic characteristics of the three groups undergoing muscle ultrasonography.

	ALS (*n* = 16)	Disease control group (*n* = 10)	Healthy control group (*n* = 10)	*P* value
Gender: male, female	11 : 5	8 : 2	6 : 4	0.531
Age	61.69 ± 7.26	45.20 ± 16.03	54.50 ± 11.81	0.024
Disease duration (months)	15.13 ± 9.70	13.80 ± 18.55	N/A	0.234
ALSFRS-R score	38.40 ± 5.75	N/A	N/A	N/A

**Table 2:** Comparison of the detection rate of muscle fasciculation among the three groups.

	ALS	Disease control group	Healthy control group	*P* value
Total fibrillation detection rate	58.50%	10.90%	4.50%	<0.001
Fasciculation muscle number	6.44 ± 2.56	1.20 ± 1.87	0.50 ± 1.08	<0.001

**Table 3:** Comparison of the fasciculation detection rate of each muscle by muscle ultrasound in the three groups.

Muscle	Detection rate of fibrillation (%)			*P* value	*P* value	*P* value
	ALS	Disease control group	Healthy control group			
Tongue muscle	18.8	0	0	0.129	0.145	0.145
Trapezius, left	37.5	0	0	0.011	0.026	0.027
Trapezius, right	43.8	0	0	0.004	0.014	0.015
Biceps, left	56.3	30.0	10.0	0.051	0.193	0.018
Biceps, right	81.3	20.0	10.0	<0.001	0.003	<0.001
Abductor pollicis brevis, left	50.0	20.0	0	0.016	0.125	0.007
Abductor pollicis brevis, right	75.0	10.0	10.0	<0.001	0.001	0.001

**Table 4:** The correlation between the detection rate of fascicular fibrillation in patients with ALS and the course of disease and ALSFRS-R.

Variable	Linear correlation coefficient (*r*)	*P*
Disease duration-fasciculation detection rate	-0.501	0.048
ALSFRS score-fasciculation detection rate	0.014	0.960

## Data Availability

The data used to support the findings of this study are available from the corresponding author upon request.
